The article "Emerging carbon-based flexible anodes for potassium-ion batteries: Progress and opportunities" was published in 2022. Journal: Front Chem.

# Emerging carbon-based flexible anodes for potassium-ion batteries: Progress and opportunities

**DOI:** 10.3389/fchem.2022.1002540

**Published:** 2022-09-08

**Authors:** Wenbin Li, Zihao Yang, Jiaxuan Zuo, Jingjing Wang, Xifei Li

**Affiliations:** ^1^ Shaanxi International Joint Research Center of Surface Technology for Energy Storage Materials, Xi’an Key Laboratory of New Energy Materials and Devices, Institute of Advanced Electrochemical Energy and School of Materials Science and Engineering, Xi’an University of Technology, Xi’an, China; ^2^ Key Laboratory of Advanced Batteries Materials for Electric Vehicles of China Petroleum and Chemical Industry Federation, Xi’an University of Technology, Xi’an, China

**Keywords:** flexible electrodes, potassium-ion battery, carbon-based substrates, heteroatom doping, metal nanoparticles

## Abstract

In recent years, carbon-based flexible anodes for potassium-ion batteries are increasingly investigated owing to the low reduction potential and abundant reserve of K and the simple preparation process of flexible electrodes. In this review, three main problems on pristine carbon-based flexible anodes are summarized: excessive volume change, repeated SEI growth, and low affinity with K^+^, which thus leads to severe capacity fade, sluggish K^+^ diffusion dynamics, and limited active sites. In this regard, the recent progress on the various modification strategies is introduced in detail, which are categorized as heteroatom-doping, coupling with metal and chalcogenide nanoparticles, and coupling with other carbonaceous materials. It is found that the doping of heteroatoms can bring the five enhancement effects of increasing active sites, improving electrical conductivity, expediting K^+^ diffusion, strengthening structural stability, and enlarging interlayer spacing. The coupling of metal and chalcogenide nanoparticles can largely offset the weakness of the scarcity of K^+^ storage sites and the poor wettability of pristine carbon-based flexible electrodes. The alloy nanoparticles consisting of the electrochemically active and inactive metals can concurrently gain a stable structure and high capacity in comparison to mono-metal nanoparticles. The coupling of the carbonaceous materials with different characteristics can coordinate the advantages of the nanostructure from graphite carbon, the defects and vacancies from amorphous carbon, and the independent structure from support carbon. Finally, the emerging challenges and opportunities for the development of carbon-based flexible anodes are presented.

## Introduction

At present, the increasing energy demand leads to the depletion of fossil fuels, deterioration of the environment, and pollution, which puts forward higher requirements for the efficient use of renewable clean energy, such as solar energy, wave energy, wind energy, and other renewable energy (Eftekhari et al., 2017). However, the intermittent characteristics and geographic selectivity limit their stable output. Developing low-cost and high-performance energy-storage systems is a feasible solution, where rechargeable batteries have attracted much attention due to their low pollution, high efficiency, and long life cycle (Hong et al., 2021; Hwang et al., 2018). As the mature and most widely used rechargeable battery, lithium-ion batteries (LIBs) have gained popular application in daily electronic products, electric vehicles, and energy-storage systems (Li et al., 2018b). However, the shortage of commercially available Li resources on Earth makes it difficult to meet the rapidly growing demand of the market, and the cost of lithium salt rapidly increases year by year, which greatly influences the development prospects of LIBs (Wang et al., 2021a; (Yang et al., 2021b). As a result, concerns about the price and depletion of lithium have accelerated the search for alternatives to LIBs in recent years (Yao and Zhu, 2020).

Potassium (K) possesses a lower reduction potential than lithium, which allows the potassium-ion batteries (PIBs) to operate at a higher potential, bringing a higher energy density (Pramudita et al., 2017). At the same time, elements of potassium are abundant on Earth and have similar chemical properties to lithium. Therefore, PIBs have received widespread attention in recent years and are regarded as a more likely alternative to LIBs (Hwang et al., 2018; (Rajagopalan et al., 2020). Generally, in a full-battery system, the anode is a key configuration that determines the electrochemical performance of the battery. The preparation process of a powder electrode for PIBs is mainly based on the slurry coating method, where the slurry mixed with the active material, conductive carbon, and adhesive in different proportions is coated on copper or aluminum foil (Wu et al., 2019b). On the one hand, during the repeated insertion and extraction of bulky K^+^ by conversion or alloying reactions, the anode material would undergo excessive volume change, thus producing severe pulverization (Xu et al., 2020), especially, the weak contact of the powder electrode material with the current collector would further result in the exfoliation of pulverized active materials, eventually leading to rapid capacity decline (Wang et al., 2020b). On the other hand, the addition of a binder and conductive carbon restricts the loading of active materials, and hence, affects the energy density of the battery. Meanwhile, the degradation of binders and the generation of side reactions through the interaction of binders and electrolytes lead to worse capacity stability during the long cycle process. In response to the aforementioned two issues of powder electrodes, the traditional slurry casting method needs to be improved or even replaced; in other words, it is necessary to search for a new type of electrode (Liu et al., 2021; (Xiong et al., 2013).

In recent years, with the increasing demand for flexible devices such as wearable devices, roll-up displays, and soft portable electronic products, there are more studies on flexible and environmentally friendly electrochemical energy-storage devices. Flexible electrodes have been raised and developed to improve the electrochemical performance of PIBs and avoid the complicated preparation process of powder electrodes (Kang et al., 2017). The independent electrode structure provides flexible properties, possesses the characteristics of non-binder and solvent-free electrode preparation, and eliminates the use of a collector during battery assembly. Meanwhile, a tightly bind of support and active electrode materials are thought to accommodate the volumetric change and the decomposition of electrode materials during battery applications. In flexible electrodes, the supports usually include the commercial carbon fiber cloth with three-dimensional structures, good flexibility, and good conductivity (Fan et al., 2022), carbon nanotubes with excellent physical, chemical, and mechanical properties (Zhao et al., 2017), nickel foam with three-dimensional uniform network structures (Huang et al., 2014), and graphene with a large surface area, high conductivity (Wu et al., 2019a), and so on.

To the best of our knowledge, there have already been several excellent reviews devoted to PIBs or flexible energy-storage devices, whereas, a comprehensive review focusing on flexible anodes for PIBs has not been reported up to now, because the application of self-supporting materials in PIBs is in its infancy. Considering this, in this review, our main contribution is to summarize and briefly discuss the recent development of flexible anodes for PIBs. Especially, the modification method of self-supporting carbon-based materials and the electrochemical enhancement mechanism of carbon-based flexible electrodes are introduced in detail. In conclusion, through this review, we aim to better understand the flexible anode materials for PIBs and provide guidance for the infancy design of non-binder potassium-based energy-storage devices in the future (Jian et al., 2016; (Jiang et al., 2020).

## Carbon-based flexible anodes for PIBS

Carbonaceous materials usually possess superior conductivity, excellent structural stability, and unique mechanics (Yang et al., 2020). Thus, abundant reported flexible electrodes are developed based on carbon-based materials (graphene films, carbon cloth, carbon nanofibers, carbon foams, etc.). When applied in PIBs, the flexible carbonaceous material can not only serve as an active material by itself but also support other active materials (Kim et al., 2018). As a result, highly flexible carbon-based materials have been extensively studied as anodes for PIBs.

Jian et al. (2015) reported for the first time that K^+^ can electrochemically intercalate into carbonaceous materials at ambient temperature and pressure. The local K^+^ insertion phenomenon between graphite layers is indicated in Figure 1A, where graphite can be reversibly intercalated by K^+^, showing a reversible capacity of 273 mAh g^−1^ at low current density. However, as the current density rises, the reversible capacity of graphite decreases sharply (Figure 1B), which may be related to the severe volume expansion of the dense graphite structure. Thereafter, carbon-based materials as the flexible materials for K^+^ storage have also been applied. Wang et al. (2021b) first synthesized an rGO film using the modified Hummer’s method and directly employed it as the PIB anode without utilizing any binder, carbon additives, and current collector (Figure 1C) (Eftekhari et al., 2017). The self-supporting electrode exhibits excellent electrochemical performance with a charge capacity of 222 mAh g^−1^ at 5 mA g^−1^, and a capacity of 150 mAh g^−1^ after 175 cycles at 10 mA g^−1^ (Figure 1D). This work presents a broader application foreground of carbonaceous materials as a PIB free-standing electrode (Luo et al., 2015).

**FIGURE 1:** **(A)** Structure diagrams of different K-GICs, side view (up) and top view (down). **(B)** Rate performance of graphite. Reproduced with permission (Jian et al., 2015). Copyright 2015, ACS. **(C)** Schematic illustration of electrochemical intercalation of K^+^ into graphite and reduced graphene oxide (RGO). **(D)** Discharge/charge profiles for graphite electrodes at various current densities. Reproduced with permission (Eftekhari et al., 2017). Copyright 2015, ACS.

However, there are three problems with the pristine carbon-based materials directly employed as the flexible anode for PIBs: excessive volume change, repeated SEI growth and low affinity with K^+^, which thus leads to severe capacity degradation, sluggish K^+^ diffusion dynamics, and limited active sites (Jing et al., 2020; (Kim et al., 2018; (Li et al., 2020). Concretely, the pristine carbonaceous materials are plagued by a resulting 61% volumetric change and the repeated SEI growth, thus bringing the fast capacity degradation and increased impedance. Meanwhile, the pristine carbonaceous materials produce a high energy barrier and low binding energy with K^+^, which thus inhibits the K^+^ diffusion through a graphene basal plane and brings the K^+^ agglomeration on the electrode surface, eventually leading to discontented electrochemical performance (Ju et al., 2016). These obstacles greatly affect the application and profound development of carbon-based flexible materials in PIBs (Ahmad et al., 2018). Therefore, to better utilize the carbon-based material as a flexible anode of PIBs, they are necessary to be further modified. Herein, combining the theoretical investigation with the experimental observation, the modification strategies of carbon-based materials and the electrochemical enhancement mechanism of carbon-based flexible anodes for PIBs are systematically discussed in the following sections.

## Modification strategies of carbon-based flexible anodes for PIBS

### Heteroatom-doping

#### Monoatom-doping

Recently, related research studies have indicated that the electrochemical performances of carbonaceous materials could be regulated and ameliorated via heteroatom doping, which has almost no influence on the intrinsic electrode structure (Li et al., 2020). The doping of the heteroatom has the ability to create defects, edges, pores, vacancies, and strained regions, and hence, can bring the five enhancement effects of increasing active sites, improving electrical conductivity, expediting K^+^ diffusion, strengthening the structural stability, and enlarging interlayer spacing. Thus, heteroatom doping contributes to elevating K^+^ storage properties, which have attracted considerable interest (Peng et al., 2020; Zhang et al., 2020). Doping of N can simultaneously provide active sites and increase electrical conductivity, and doping of S can induce more active sites (Hong et al., 2018; Park et al., 2022). Wang et al. (2021b) synthesized 6.3 wt% N-doped flexible biomass carbon membranes by employing the C source of chitosan (CS, Figure 2A). The faveolate construction contributes to improving the e^−^ transfer ability (Figures 2B,C). Meanwhile, the first principle DFT calculation demonstrates that the pyridine N observably enhances the adsorption capacity of carbonaceous materials for K^+^. Thus, the flexible N-doped CS-derived carbon membrane electrode displays an excellent rate capability and a stable capacity of 146 mAh g^−1^ at 2 A g^−1^ after 500 cycles. Except for N-doping, Li et al. (2018a) designed 10.17 wt% S-doped reduced graphene oxide sponge (S-RGO) flexible electrode via freeze-drying of GO solution and a further calcination operation in a S gas atmosphere (Figure 2D). Different from the role of N, the introduction of S triggers more active sites on the electrode surface, hence facilitating the K^+^ transfer, increasing the K^+^ storage sites, strengthening the structural stability, and extending the cycling life (Wu et al., 2019b). As a result, the S-RGO flexible electrode delivers a high capacity of 229 mAh g^−1^ after 500 cycles at 1 A g^−1^.

**FIGURE 2:** **(A)** Schematic representation of the preparation process of a flexible CS-derived carbon membrane. **(B,C)** Illustration of the storage mechanism of K^+^ in the porous CS-derived carbon membrane. Reproduced with permission (Wang et al., 2021b). Copyright 2021 Elsevier Ltd. **(D)** Possible K^+^ storage mechanism for S-RGO sponges. Reproduced with permission (Li et al., 2018a). Copyright 2019 Wiley-VCH.

The characterization of graphene could be changed when a single element is doped into graphene sheets, which thus exhibits enhanced electronic conductivity (An et al., 2019). Nevertheless, the electrochemical performance of carbon-based flexible electrodes is still not completely manifested. One main reason is the barriers to e^−^ transport and ion diffusion in the cross-plane direction, once carbonaceous materials have been tightly restacked to form the film structure (Adams et al., 2019). Another reason is that the absence of long-range order in the hard-carbon electrode decreases the electrical conductivity, and the electrode generally shows an inconspicuous plateau for K^+^ storage, thus leading to a low energy density of the full cell when paired with cathode materials (Zeng et al., 2020). Therefore, to prepare high-performance PIB anode materials, the focus should be shifted to synergistic enhancement (Li et al., 2014).

#### Dual-doping

To overcome the weaknesses of monoatom-doping, a dual-doping strategy is developed to synergize the effect of each specie in boosting the electrochemical performances of carbonaceous materials (Tao et al., 2020). Recently, the as-reported works on the dual-doping of carbonaceous materials involve a N, O dual-doped hard carbon anode (Adams et al., 2017; Gong et al., 2019), P, N dual-doped carbon (Gan et al., 2019), P, O dual-doped graphene (Zhao et al., 2021), and so on. The dual-doping strategy has been also used on flexible carbon-based substrates in consideration of its synergistic effect on the electrode surface (Liu et al., 2022). Zeng et al. (2020) designed flexible a N, O dual-doped carbon-coated graphene foam film (NOC@GF), where the N, O doped hard carbon layer boosts K^+^ adsorption and the graphene layer shows a low resistance for K^+^ diffusion (Figure 3A). The NOC@GF anode displays a large capacity of 281 mAh g^−1^ at 1 A g^−1^ after 5,500 cycles (Figure 3B) and shows excellent rate capability with a reversible capacity of 123 mAh g^−1^ at 5.0 A g^−1^ Figure 3C). When the current density is tuned back to 0.1 A g^−1^, the specific capacity can still reach 341 mAh g^−1^. This excellent electrochemical performance can be attributed to the subtle doping of N and O, which promotes the adsorption of K^+^, leads to excellent pseudo capacitance behavior, and makes the graphene layer have a low K^+^ diffusion barrier. This hybrid nanostructure provides a new promising approach to developing high-performance flexible carbon-based K^+^ storage anodes.

**FIGURE 3:** **(A)** Theoretical simulations of K-atom adsorption and diffusion. **(B)** Cycling performances at 1 A g^−1^ and **(C)** rate performances at the current densities from 0.1 to 5 A g^−1^ for NOC@GF and the NOC-F anode. Reproduced with permission (Zeng et al., 2020). Copyright 2021 Elsevier Ltd. **(D)** Preparation diagram and **(E)** cycling performances at various current densities for the N, P-VG@CC anode. Reproduced with permission (Qiu et al., 2019). Copyright 2019 WILEY-VCH.

Qiu et al. (2019) prepared N and P dual-doped vertical graphene (VG) arrays on carbon clothes (N, P-VG@CC) as a flexible anode of PIBs (Figure 3D). Benefiting from the large surface of carbon clothes, the abundant active sites and enhanced ionic conductivity caused by N, P dual-doping and the enlarged interlayer distance, the N, P-VG@CC flexible electrode presents a remarkable cycling and rate performance, as shown in Figure 3E. At a low current density (25 mA g^−1^), the electrode shows a high reversible capacity (342.9 mAh g^−1^). After 1,000 cycles, the electrode still maintains a reversible capacity of 281.1 mAh g^−1^ with a capacity retention of 82%. Afterward, Gong et al. (2021) proposed a supercritical CO_2_ foaming and pyrolysis technology to fabricate a N, O dual-doped Bi-continuous carbon scaffold (BNCS). The N, O dual-doping and defective nature of amorphous carbon trigger plenty of accessible active sites for K^+^ storage. Thus, the N/O dual-doped BNCS anode for PIBs performs a large capacity of 325 mAh g^−1^ after 300 cycles at 0.1 A g^−1^, superior rate performance with a capacity of 118 mAh g^−1^ at 10 A g^−1^, and ultra-long cycling performance with a capacity of 184 mAh g^−1^ after 5,000 cycles at 1 A g^−1^.

### Coupling with metal and chalcogenide nanoparticles

According to the theoretical calculation, the metal nanoparticles composed of group IVA and VA elements, such as Co (Yang et al., 2021a), Sb (Guan et al., 2019), Sn (Jiang et al., 2019), Bi (Wang et al., 2020a), and the metal chalcogenide nanoparticles, such as Fe_2_O_3_ (Sultana et al., 2017), MoSSe (Tian et al., 2020c), and Sb_2_Se_3_ (Yang et al., 2022), have higher K^+^ storage capacity than carbonaceous materials owing to their polymerous conversion and alloying reaction (Yuan et al., 2021). Thus, the coupling of metal and chalcogenide nanoparticles can largely offset the weakness of the scarcity of K^+^ storage sites and the poor wettability of the pristine carbon-based flexible electrode. However, the larger radius of K^+^ makes it difficult to buffer the intensive stress produced by active materials and suppress the volume expansion during the insertion/extraction process, thus leading to rapid capacity fading upon cycling (Mao et al., 2018). So far, researchers have tried to solve these inherent problems of metal and chalcogenide nanoparticle anodes (Wu et al., 2021a; Zheng et al., 2020). By combining the high specific capacity of metal and chalcogenides with the stable structure of various carbonaceous materials, the carbon-based composite anode can simultaneously alleviate the volume expansion and increase the K^+^ storage capacity to a large extent (Wu et al., 2021b).

#### Coupling with mono-metal nanoparticles

Metallic Sb possessing high theoretical capacity (K_3_Sb, 660 mAh g^−1^), small electrochemical polarization (0.2 V), and low operating voltage has been broadly investigated as one of the potential PIB anode materials (Wu et al., 2021c). However, the huge volume change upon cycling easily causes electrode degradation, leading to poor rate capability and cycling stability. For this reason, Sb nanoparticles encapsulated in N, P dual-doped mesoporous carbon nanofibers (Sb@NPMC) were fabricated by Zhang et al. (2018). The unique structure presents superior electrical conductivity between Sb nanoparticles and carbon nanofibers matrix and accommodates the volume change of Sb nanoparticles. Unfortunately, the usage of a binder in the Sb@NPMC powder anode gives rise to unsatisfactory rate performance and cycle capacity. Therefore, coupling the carbonaceous materials with mono-metal Sb nanoparticles to serve as a self-supporting electrode is a potential strategy to solve the aforementioned problem. Ge et al. (2019) designed and prepared *in situ* encapsulating ultrafine Sb nanocrystals within carbon nanofibers composed of an array of nanochannels (u-Sb@CNFs) as a flexible PIB anode. As shown in the synthetic route of the u-Sb@CNF flexible electrode in Figure 4A, the Sb ultrafine nanocrystals are evenly embedded in the multi-nanochannels containing CNFs, and each nanofiber contains an inbuilt polystyrene nanofiber array carrying Sb^3+^. The ultrafine nanostructures and hollow nanochannels can enable fast K^+^ migration and strain relaxation. As a result, the u-Sb@CNF free-standing electrode manifests excellent cycling performance with a capacity of 459 mAh g^−1^ over 100 cycles at 0.2 A g^−1^ (Figure 4B).

**FIGURE 4:** **(A)** Preparation diagram of the u-Sb@CNF free-standing electrode. **(B)** Rate properties of u-Sb@CNFs and Sb@s-CNFs. Reproduced with permission (Ge et al., 2019). Copyright 2019 WILEY-VCH. **(C)** SEM and **(D)** HRTEM images of Sb-G-C. **(E)** Schematic of the mixed K^+^ storage mechanism of Sb-G-C nanofibers. Reproduced with permission. (Huang et al., 2021). Copyright 2021 ESC.

Subsequently, Huang et al. (2021) fabricated porous Sb–graphene–carbon nanofibers through an electrospinning technique (Sb-G-C, Figures 4C,D). The compatible Sb/nanofiber interface effectively strengthens the cycling ability. Meanwhile, the dispersive graphene provides moderate cushioning to tolerate K^+^ storage, and thus, inhibits volume expansion, creates more open transfer routes, and accelerates the charge transport. In addition, they further proposed that there are three kinds of K^+^ storage sites: defect or edge, micro-pore, and interlamination (Figure 4E). Thus, the Sb-G-C flexible anode shows superior cycling performance with a capacity of 205 mAh g^−1^ after 100 cycles at 0.1 A g^−1^ and outstanding rate performance with a capacity of 121 mAh g^−1^ at 1 A g^−1^. The main problem faced by alloy anode materials for PIBs is the serious volume effect, and the electrochemical performance has been improved by means of combining with carbon materials. However, for single-metal composite materials, the proportion of carbonaceous materials in self-supporting materials is usually higher, which will reduce the specific capacity of the whole battery, and thus, mask the advantages of alloy anode materials. Therefore, it is necessary to appropriately increase the proportion of metals.

#### Coupling with alloy nanoparticles

In addition to mono-metal nanoparticles, many research studies have also shown that alloy nanoparticles have more K^+^ storage sites than the intercalated anode (Cao et al., 2021). Especially, the alloy nanoparticles consisting of electrochemically active and inactive metals can concurrently attain high capacity and stable structure in comparison to mono-metal nanoparticles (Qi et al., 2020). For example, Han et al. (2019) synthesized a kind of N-doped CoSb@C nanofiber (Figure 5A), where plentiful CoSb nanoparticles are evenly embedded in the carbon nanofiber possessing a diameter of ∼200 nm for the pristine anode material (Figure 5B). In the CoSb alloy, the metal Co, as an electrochemically inactive metal, significantly inhibits the carbide phase transition, presents a buffer for excessive volume expansion, and induces the generation of steady SEI. Meanwhile, metal Sb with high theoretical capacity can provide plentiful active sites for K^+^ storage.

**FIGURE 5:** **(A)** Schematic diagram of the electrochemical enhancement mechanism of CoSb@C nanofibers. **(B–D)** SEM images of CoSb@C nanofibers during the initial cycle process. **(E)** Rate performance and **(F)** long-term K^+^ storage performance of CoSb@C nanofibers’ electrode at 1 A g^−1^. Reproduced with permission (Han et al., 2019). Copyright 2019 RSC.

The structural evolution of N-doped CoSb@C nanofibers at different voltages demonstrates that the surface of nanofibers becomes smooth after initially discharging to 0.01 V (Figure 5C), which is caused by the thorough conversion of Sb to K_3_Sb. When the voltage is returned to 3.0 V, CoSb nanoparticles are regenerated (Figure 5D), suggesting the structure stability and the reversibility of the electrochemical reaction. Thus, the bimetallic CoSb alloys can be applied as a high-capacity flexible anode for PIBs, where a large cycling capacity of 250 mAh g^−1^ at 1 A g^−1^ after 500 cycles is gained and a superior rate capacity of 160 mA h g^−1^ at 2 A g^−1^ is realized (Figures 5E,F). After that, the work of bimetallic compatible flexible anodes has also been reported by Xue et al. (2021). They synthesized hollow CoSn alloy nanoboxes (Figures 6A–C) embedded inside N-doped C nanotubes (CoSn@N-C (Figures 6D–F) by the synthesis technique shown in Figure 6G.

**FIGURE 6:** **(A)** TEM image, **(B)** HRTEM image, and **(C)** SAED pattern of CoSn(OH)_6_ nanoboxes. **(D)** TEM image, **(E)** HRTEM image, and **(F)** SAED pattern of CoSn@N-C nanotubes. **(G)** Synthesis diagram of CoSn@N-C nanotubes. Reproduced with permission (Xue et al., 2021). Copyright 2021 Elsevier Ltd.

When employed as the flexible anode for PIBs, CoSn@N-C nanotubes have three advantages. First, the inactive metal Co matrix and the holes in the nanoboxes ensure the effective mitigation of the stress caused by excessive Sn volume expansion. Second, the encapsulation layer of nanotubes prevents the fracture of nanoboxes during the repeated insertion/extraction of K^+^ and accelerates the infiltration of the electrolyte into the electrode material and hence promotes the electrochemical dynamics. Third, the CoSn@N-C membrane can be directly employed as a flexible PIB anode in the premise of no binder and current collector, which contributes to obtaining great energy density. Benefitting from the aforementioned three advantages, the CoSn@N-C flexible anode delivers a large capacity of 178 mAh g^−1^ after 2,000 cycles at 0.5 A g^−1^ and superior rate capacity of 134.8 mAh g^−1^ at 10 A g^−1^.

Alloy nanoparticles’ anode materials often exhibit higher theoretical specific capacity. Especially, when two kinds of metal with electrochemical activity form alloys, they can exploit their respective advantages for potassium storage. When the carbon-based self-supporting materials are combined with the aforementioned alloy nanoparticles, the cycle stability can be improved to a certain extent, but it is still necessary to cooperate with the regulation of the structure and specific surface area to further enhance the electrochemical performance.

#### Coupling with metal chalcogenide nanoparticles

During the latest decade, metal chalcogenides have attracted increasing attention and developed rapidly as a kind of hot research material in the energy storage and conversion field. In the as-reported PIBs, metal chalcogenides are commonly composed of metals such as Mo, Fe, Sb, Co, and V and chalcogens O, S, and Se. However, in the K^+^ storage process, these electrodes manifest poor cycling performance and weak rate capability due to their serious volume fluctuations, low electron and ionic conductivity, and big K^+^ radius. Among various solution strategies, it is an effective strategy to introduce flexible carbon-based materials to restrain the excessive volume expansion and quicken e^−^ transfer. Tian et al. (2020b) prepared a flexible anode composed of the MoSSe arrays with dual anionic vacancies and a carbon nanofiber membrane (v-MoSSe@CM, Figures 7A,B). The 3D framework of carbon nanofibers suppresses the agglomeration of MoSSe nanosheets and relieves excessive volume change, and hence decreases the possibility of nano-construction collapse during the repeated K^+^ insertion/extraction process. Benefiting from these advantages, the flexible v-MoSSe@CM anode demonstrates an excellent rate performance (202 mAh g^−1^ at 5 A g^−1^) and superior cycling performance (220.5 mAh g^−1^ at 0.5 A g^−1^ after 1,000 cycles, Figure 7C).

**FIGURE 7:** **(A)** SEM and **(B)** elemental mapping images of v-MoSSe@CM. **(C)** Second, 10^th^, and 200th charge/discharge profiles at 0.5 A g^−1^ for v-MoSSe@CM. Reproduced with permission (Tian et al., 2020b). Copyright 2021 Elsevier Ltd. Schematic of K^+^ transport kinetics in **(D)** G (0.375 nm), **(E)** G (0.407 nm), and **(F)** OM-G-400 (0.407 nm) anodes at different discharging times. **(G)** Cycling performance of 2,000 cycles at 1 A g^−1^ and **(H)** rate performance for OM-G and G-400 anodes. Reproduced with permission (Qiao et al., 2021). Copyright 2021 WILEY-VCH.

In addition, the precise control of the material microstructure at the molecular and nanoscale is also pivotal to enhancing the electrochemical performance and discovering differentiated energy storage mechanisms. For example, Qiao et al. (2021) proposed a self-growing strategy to synchronously regulate the interlayer distance and hydrophilicity of graphene layers and, hence, set up neoteric graphene structures possessing super high K^+^ storage ability. On the surface of the unique graphene, the ultrafine Fe_2_O_3_ nanoclusters/nanoparticles are *in situ* bonded with graphene. Furthermore, the interlayer distance is enlarged from 0.375 to 0.407 nm through the fine regulation of Fe_2_O_3_ nanoparticles as nanorods (Figures 7D–F). The aforementioned two structural features contribute to affording a big space for K^+^ storage and relieving the excessive volume change during K^+^ insertion/extraction process. Meanwhile, Fe_2_O_3_ nanoparticles improve the hydrophilicity of graphene to electrolyte, and hence accelerate the infiltration and retainability of the electrolyte in the graphene. As a result, the flexible anode demonstrates significantly enhanced K^+^ storage properties (Figures 7G,H). The capacity arrives at 496.4 and 306.6 mAh g^−1^ at 0.1 and 10 A g^−1^, respectively. After cycling 2,000 times at 1 A g^−1^, the capacity retention can reach 96.3%.

For Sb-based metal chalcogenides, the alloying reaction provides the main capacity. However, the shortcomings of the large radius of K^+^ and the sluggish reaction kinetics in the alloying process affect the cyclic stability. In this regard, we used vacuum filtration and a subsequent annealing process to construct the Sb_2_Se_3_ nanorods on the surface of graphene (Sb_2_Se_3_@h-rGO) with the formation of Sb-O-C chemical bonds in their interfaces in the previous work (Figures 8A,B) (Yang et al., 2022). These as-constructed chemical bonds can effectively reduce the diffusion energy barrier of K^+^ in the de-alloying reaction, promoting the formation/breaking of K-Sb bonds in the discharge alloy product of K_3_Sb. Therefore, Sb_2_Se_3_@h-rGO shows excellent electrochemical performance when used as a free-standing anode for PIBs.

**FIGURE 8:** K diffusion paths in **(A)** K_3_Sb@graphene and **(B)** K_3_Sb model. **(C)** Rate capability for free-standing Sb_2_Se_3_@h-rGO electrodes. SEM images of **(D)** free-standing Sb_2_Se_3_@h-rGO electrode and **(E)** Sb_2_Se_3_ powder electrode after 50 repeated cycles. **(F)** Cycling performances of the free-standing Sb_2_Se_3_@h-rGO electrode at 0.1 A g^−1^ for 500 cycles. Reproduced with permission (Yang et al., 2022). Copyright 2021 Elsevier Ltd.

The specific capacity of Sb_2_Se_3_@h-rGO arrives at 73 mAh g^−1^ at the current density of 2 A g^−1^ (Figure 8C). After 50 cycles at 0.1 A g^−1^, the nanorod morphology is well maintained (Figures 8D,E), suggesting its outstanding microstructure reversibility. After 500 cycles, the free-standing electrode can still deliver the specific capacity of 382 mAh g^−1^ at 0.1 A g^−1^ (Figure 8F). In addition to the aforementioned reports, many other free-standing electrodes composed of metal chalcogenide such as SnO_2_ (Qiu et al., 2020) and V_2_O_3_ (Jin et al., 2018) with carbon-based materials have also been reported, and have excellent electrochemical properties.

### Coupling with other carbonaceous materials

Carbonaceous materials with narrow interlayer spacing frequently show poor circulation ability as PIB anodes on account of the large volume change and further structure collapse induced by the repeated insertion of K^+^. The coupling of the carbonaceous materials with different characteristics is conducive to gathering the preponderances of the nanostructure from graphite carbon, the defects and vacancies from amorphous carbon, and the independent structure from matrix carbon (Liu et al., 2018).

Thus, the abundant K^+^ storage sites, stable cycle structure, and fast charge transfer can be realized simultaneously for the flexible carbon-based composite electrode. For example, Tian et al. (2020a) reported highly graphitized carbon nanofibers (HG-CNFs) as a free-standing anode for PIBs. Different from other carbon-based materials (Figures 9A,B), the interconnected network and large interlayer spacing in the HG-CNF flexible electrode alleviate the excessive volume change and thus reinforce the structural stability of the electrode. For this reason, the HG-CNF flexible anode delivers an outstanding K^+^ storage capacity of 264.4 mAh g^−1^ with a stable plateau voltage below 0.2 V and superior cycling stability with a very small capacity degradation of 0.008% per cycle at 56 mA g^−1^ after 400 cycles (Figures 9C,D).

**FIGURE 9:** **(A)** HRTEM image of graphitic. **(B)** Digital photograph of folded HG-CNFs. **(C)** Rate capabilities from 0.1 to 35 C for LG-CNFs and HG-CNFs. **(D)** Long-term cycle stability and corresponding Coulombic efficiency of HG-CNFs at 0.2 C. Reproduced with permission (Tian et al., 2020b). Copyright 2020 Elsevier Ltd.

Shen et al. (2019) prepared free-standing carbon nanotubes encapsulated in a sub-micro carbon fiber (SMCF@CNTs, Figure 10A) as the PIB anode. The introduction of CNTs simultaneously upgrades the capacitive and diffusion-controlled K^+^ storage, where the capacitance contribution arrives at more than 60%. Thus, the flexible SMCF@CNTs anode demonstrates excellent K^+^ storage property with a rate capacity of 108 mAh g^−1^ at 135.9 mAh g^−1^ (Figure 10B) and a durable cycling life with a capacity of 193 mAh g^−1^ after 300 times at 279 mAh g^−1^ (Figure 10C). Zeng et al. (2019) constructed carbon nanotubes on the graphitic carbon foam with 3D porous interconnected nanoarchitecture (CNTs/GCF, Figure 10D). Benefiting from the superior e^−^ transfer ability of CNTs, the CNT/GCF film shows low interfacial resistance and rapid K^+^ diffusion. At the same time, the porous GCF possessing a 3D pipeline frame shows a stable structure and enables the electrolyte to infiltrate the electrode, eventually affording unobstructed K^+^ transfer channels. As a result, the flexible anode delivers reversible capacities of 254, 233, 204, 113, 85, and 74 mAh g^−1^ at the current densities of 0.05, 0.1 0.2, 0.5, 0.8, and 1.0 A g^−1^, respectively, and a stable and low-discharge platform can be obtained (Figure 10E). It also demonstrates superior long-term cycling performance with a capacity of 127 mAh g^−1^ at 0.5 A g^−1^ after 2,000 times (Figure 10F).

**FIGURE 10:** **(A)** TEM image of SMCF@CNTs. **(B)** Rate performance from 0.1 to 5 C. **(C)** Cycling performance at 1 C. Reproduced with permission (Shen et al., 2019). Copyright 2019 ACS. **(D)** Fabrication diagram of CNTs/GCF. **(E)** Voltage profiles at 0.1 A g^−1^ and **(F)** long-term cycle performance at 0.5 A g^−1^ for CNTs/GCF. Reproduced with permission (Zeng et al., 2019). Copyright 2019 RCS.

## Conclusion and perspectives

### Conclusion

In most cases, binder-free electrode materials often show excellent electrochemical performance such as high capacity, rate capability, and cycling stability. The electrochemical properties of the materials involved in this work are shown in Table 1. However, there are three problems with the pristine carbon-based materials directly employed as the flexible anode for PIBs: excessive volume change, rrepeated SEI growth and low affinity with K+, which thus leads to severe capacity fade, sluggish K+ diffusion dynamics and limited active sites.

**TABLE 1:** Electrochemical performance of the various carbon-based flexible anodes in the study for PIBs.

Flexible materials	Material varieties	Templates	Rate capability (mAh g^−1^)	Cyclability (mAh g^−1^)	Reference
Graphite	-	Free	80 at 279 mA g^−1^	100 at 0.14 A g^−1^ after 50 cycles	Jian et al. (2015)
rGO film	-	Free	222 at 5 mA g^−1^	150 at 0.01 A g^−1^ after 175	Luo et al. (2015)
CNF	Porous carbon nanofiber	Carbon nanofiber paper	100 at 7.7 A g^−1^	270 at 0.2 A g^−1^ after 1,200	Zhao et al. (2017)
CS	N-doped carbon	Free	-	146 at 2 A g^−1^ after 500	Wang et al. (2021b)
S-RGO	S-doped carbon	Free	361 at 50 mA g^−1^	229 at 1 A g^−1^ after 500	Li et al. (2018a)
NOC@GF	N, O dual-doped	Graphene foam	123 at 5 A g^−1^	281 at 1 A g^−1^ after 5,500	Zeng et al. (2020)
NO/CNFs	N, O dual-doped	Free	110 at 2.7 A g^−1^	170 at 0.27 A g^−1^ after 1,900	Adams et al. (2017)
N, P-VG@CC	N, P dual-doped	Carbon clothes	156.1 at 2 A g^−1^	142.4 at 1 A g^−1^ after 1,000	Qiu et al. (2019)
BNCS	N, O dual-doped	Carbon scaffold	118 at 10 A g^−1^	184 at 1 A g^−1^after 5,000	Gong et al. (2021)
u-Sb@CNFs	Sb-embedded CNFs	Free	184 at 2 A g^−1^	188 at 2 A g^−1^ after 3,000	Ge et al. (2019)
Sb-G-C	Sb-graphene-carbon	Free	120.83 at 1 A g^−1^	204.95 at 0.1 A g^−1^ after 100	Huang et al. (2021)
CoSb@C	Co, Sb-embedded CNFs	Free	160 at 2 A g^−1^	250 at 1 A g^−1^ after 500	Han et al. (2019)
CoSn@N-C	CoSn alloy-embedded CNFs	Free	134.8 at 10 A g^−1^	178 at 0.5 A g^−1^ after 2,000	Xue et al. (2021)
SnO_2_@CF	SnO_2_ grown on GF	Graphene foam	143.5 at 5 A g^−1^	231.7 at 1 A g^−1^ after 400	Qiu et al. (2020)
V_2_O_3_@PNCNFs	V_2_O_3_-embedded CNFs	Free	134 at 1 A g^−1^	240 at 0.5 A g^−1^ after 500	Jin et al. (2018)
v-MoSSe@CM	MoSSe grown on carbon	Free	202 at 5 A g^−1^	220.5 at 0.5 A g^−1^ after 1,000	Tian et al. (2020b)
OM-G	Fe_2_O_3_ bonds with graphene	Free	306.6 at 10 A g^−1^	384.8 at 1 A g^−1^ after 2,000	Qiao et al. (2021)
Sb_2_Se_3_@h-rGO	Sb_2_Se_3_ bonds with graphene	Free	73 at 2 A g^−1^	382 at 0.1 A g^−1^ after 500	Yang et al. (2022)
CDs@rGO	Carbon dots and graphene	Free	185 at 0.5 A g^−1^	244 at 0.2 A g^−1^ after 840	Liu et al. (2018)
HG-CNFs	Highly graphitized carbon	Carbon scaffold	225.7 at 9.7 A g^−1^	162.5 at 0.05 A g^−1^ after 500	Tian et al. (2020a)
SMCF@CNTs	Carbon nanotubes and fiber	Free	108 at 136 mA g^−1^	193 at 0.279 A g^−1^ after 300	Shen et al. (2019)
CNTs/GCF	Carbon nanotubes and GCF	Graphene foam	74 at 1 A g^−1^	127 at 0.5 A g^−1^ after 2,000	Zeng et al. (2019)

The modification strategies are categorized as heteroatom-doping (monoatom-doping and dual-doping), coupling with metal (mono-metal and alloy nanoparticles) and chalcogenide nanoparticles, and coupling with other carbonaceous materials. The doping of the heteroatom can bring the five enhancement effects of increasing active sites, improving electrical conductivity, expediting K^+^ diffusion, strengthening structural stability, and enlarging interlayer spacing. The coupling of metal and chalcogenide nanoparticles can largely offset the weakness of the scarcity of K^+^ storage sites and the poor wettability of pristine carbon-based flexible electrode. The alloy nanoparticles consisting of electrochemically active and inactive metals can concurrently attain a stable structure and high capacity in comparison to mono-metal nanoparticles. The coupling of the carbonaceous materials with different characteristics can coordinate the advantages of the nanostructure from graphite carbon, the defects and vacancies from amorphous carbon, and the independent structure from the support carbon.

### Perspectives

Although some investigates have been performed in the past decade, some problems and challenges still need to be solved in the practical application of carbon-based flexible anodes for PIBs:

1) More varieties of non-metallic elements, such as I, B, and Br, can be introduced, and accurately adjusting the doping element content can be carried out to further improve the K^+^ storage properties of carbon-based flexible electrodes.
2) More varieties of metal and inorganic nanoparticles with more K^+^ storage sites and better electrochemical reversibility can be coupled, and accurately adjusting the proportion of nanoparticles in the carbon-based flexible electrodes can be further explored. Especially, the hetero-interfaces between carbonaceous materials and nanoparticles need to be emphatically concerned.
3) The carbon-based substrates concurrently possessing strong mechanical properties (flexibility, tensility, and compressibility) need to be developed to further promote the application of carbon-based flexible PIB electrodes in the field of wearable devices, roll-up displays, and soft portable electronic products.
